# Protective Effect of Methylxanthine Fractions Isolated from *Bancha* Tea Leaves against Doxorubicin-Induced Cardio- and Nephrotoxicities in Rats

**DOI:** 10.1155/2020/4018412

**Published:** 2020-08-11

**Authors:** Maya P. Radeva-Ilieva, Kaloyan D. Georgiev, Nadezhda R. Hvarchanova, Stanila S. Stoeva, Iliya J. Slavov, Deyan L. Dzhenkov, Marieta P. Georgieva

**Affiliations:** ^1^Department of Pharmacology, Toxicology and Pharmacotherapy, Faculty of Pharmacy, Medical University “Prof. Dr. Paraskev Stoyanov”, Varna 9000, Bulgaria; ^2^Department of Biology, Faculty of Pharmacy, Medical University “Prof. Dr. Paraskev Stoyanov”, Varna 9000, Bulgaria; ^3^Department of General and Clinical Pathology, Forensic Medicine and Deontology, Division of General and Clinical Pathology, Faculty of Medicine, Medical University “Prof. Dr. Paraskev Stoyanov”, Varna 9000, Bulgaria

## Abstract

*Doxorubicin* is an anthracycline antibiotic that is used for the treatment of various types of cancer. However, its clinical usage is limited due to its potential life-threatening adverse effects, such as cardio- and nephrotoxicities. Nonetheless, simultaneous administration of *doxorubicin* and antioxidants, such as those found in *green tea* leaves, could reduce cardiac and renal tissue damage caused by oxidative stress. The methylxanthine fraction isolated from *Bancha tea* leaves were tested *in vitro* for its antioxidant activity and *in vivo* for its organoprotective properties against *doxorubicin*-induced cardio- and nephrotoxicities in a rat model. The *in vivo* study was conducted on male Wistar rats divided into 6 groups. Methylxanthines were administered at high (5 mg/kg body weight) and low (1 mg/kg body weight) doses, while doxorubicin was administered at a cumulative dose of 20 mg/kg body weight. Serum creatinine, uric acid, and urea concentrations, as well as serum enzyme levels (creatinine kinase (CK), creatinine kinase MB fraction (CK-MB), aspartate aminotransferase (AST), and lactate dehydrogenase (LDH)) and electrolytes (Na^+^, K^+^, and Cl^−^), were analysed. In addition, histological analysis was performed to assess cardiac and renal tissue damage. The concomitant administration of *Bancha* methylxanthines and *doxorubicin* showed a dose-dependent reduction in the serum biochemical parameters, indicating a decrease in the cardiac and renal tissue damage caused by the antibiotic. Histological analysis showed that pretreatment with methylxanthines at the dose of 5 mg/kg resulted in an almost normal myocardial structure and a significant decrease in the morphological kidney changes caused by *doxorubicin* exposure compared with the group that received *doxorubicin* alone. The putative mechanism is most likely related to a reduction in the oxidative stress caused by doxorubicin.

## 1. Introduction

*Doxorubicin* is an anthracycline antibiotic that is used for the treatment of a variety of cancer diseases, such as Hodgkin's and non-Hodgkin's lymphoma, multiple myeloma, and breast, lung, and ovarian tumours. This antibiotic is often combined with other chemotherapeutic drugs. Two major mechanisms have been proposed for the antitumour activity of *doxorubicin*. One is associated with the intercalation into DNA and inhibition of topoisomerase II progression and activity. Topoisomerase II is an essential enzyme for DNA replication, which relaxes DNA supercoils. This results in an inhibition of macromolecule biosynthesis in tumour cells. The other mechanism of action of *doxorubicin* is due to the formation of free radicals. Reductive conversion of *doxorubicin* into a semiquinone radical is essential for the cytotoxic effects. The semiquinone radical can exert direct cytotoxic effects or be oxidized back to *doxorubicin* (i.e., redox cycling), resulting in the generation of reactive oxygen species (ROS). Free radicals can lead to oxidative stress, lipid peroxidation, membrane damage, DNA damage, the induction of apoptosis, and cell death [1–4].

Dose-dependent cardio- and nephrotoxicities are some of the main serious adverse effects of *doxorubicin* treatment and are the major limiting factors for its clinical usage. *Doxorubicin*-induced cardiac and renal toxicities may be the reason for discontinuation of the therapy in some patients. This may reduce the effectiveness of antitumour therapy and worsen the condition of the patient. According to a number of studies, several mechanisms have been proposed to be responsible for the toxic effects of *doxorubicin*. In general, these mechanisms include an elevation of ROS production, which leads to oxidative stress and endothelial cell injury; an increase in intracellular iron; a decrease in antioxidant capacity of the cell; and an activation of the apoptotic cascade. Therefore, it can be assumed that the simultaneous administration of antioxidants and *doxorubicin* could lead to a reduction in cardiac and renal tissue damage related to oxidative stress [5–9].

*Green tea* is famous worldwide for its antioxidative properties. It is made from the leaves of *Camellia sinensis* (*L.*) *Kuntze*, *Theaceae*. Green tea consumption is an important part of Chinese and Japanese traditional cultures. There are different types of green tea depending on the manufacturing process, which determines the difference in the quantity of the bioactive compounds. Some of the most common types of green tea in Japan are *Sencha* and *Bancha*. *Sencha* is the first or second flush of green tea (first seasonal picking), while *Bancha* is the third or fourth flush of green tea (late seasonal picking) [10].

Green tea contains bioactive ingredients such as polyphenols and methylxanthines. Polyphenols have been widely studied for their diverse pharmacological effects. The most researched methylxanthines are *caffeine*, *theophylline*, and *theobromine*. These compounds are purine alkaloids that naturally occur in coffee, tea leaves, cocoa beans, and other substances. *Caffeine* is the most widespread and consumed methylxanthine, and it is classified as a stimulant of the central nervous system and the cardiovascular system. *Theophylline* acts as a bronchodilator, while *theobromine* relaxes blood vessels, decreases blood pressure, and increases heart rate [11, 12].

The objective of the present study was to evaluate the antioxidant activity *in vitro* and the potential protective effects of methylxanthine fractions isolated from *Bancha* tea leaves *in vivo* against doxorubicin-induced cardio- and nephrotoxicities in rats.

## 2. Materials and Methods

### 2.1. Animals

The study was performed on 36 male Wistar rats weighing 180-200 g. The animals were obtained from the Medical University of Varna, Bulgaria. The animals were housed in a well-ventilated room on a 12 h light/dark cycle with free access to standard rat chow and water. The temperature was maintained at 23 ± 2°C, and the humidity was 50 ± 10%. All experimental procedures were performed between 8 and 10 a.m. The study was conducted according to the national requirements for the protection and humane treatment of laboratory animals, complying with the European Communities Council Directives 86/609/EEC. For the performed experimental procedures, permission was obtained from the Bulgarian Food Safety Agency (BFSA).

### 2.2. Chemicals

*Doxorubicin* (DOX) was obtained as *doxorubicin hydrochloride*, a concentrate for solution for infusion (2 mg/mL) from Accord Healthcare Limited, United Kingdom. *Bancha* tea leaves were purchased from a local market with quality assurance, and the material was stored at room temperature. They were pharmacognostically identified by Assoc. Prof. Iliya Slavov from the Department of Biology, Sector Pharmaceutical Botany and Pharmacognosy, Faculty of Pharmacy, Medical University of Varna, Bulgaria. The extraction conditions and high-performance liquid chromatography (HPLC) analysis of the methylxanthine fraction were described in detail in a previous study [13].

### 2.3. Assessment of Antioxidant Activity (AA)

#### 2.3.1. 2,2-Diphenyl-1-picrylhydrazyl (DPPH) Free-Radical Scavenging Activity

The method was performed according to Brand-Williams et al. [14] with slight modifications. A freshly prepared 4 × 10^−4^ M methanolic solution of DPPH was mixed with the samples in a ratio of 2 : 0.5 (*v*/*v*). The light absorption was measured at 517 nm. The DPPH radical scavenging activity was presented as a function of the concentration of trolox (trolox equivalent antioxidant capacity (TEAC)) and was defined as the concentration of trolox having an equivalent AA, expressed as *μ*M/trolox equivalent (TE) gram dry extract (DE).

#### 2.3.2. 2,2′-Azino-bis-(3-ethylbenzothiazoline-6-sulfonic Acid) (ABTS) Cation Decolourization Assay

This method was conducted as described by Georgiev et al. [13]. Briefly, ABTS was dissolved to a concentration of 7 mM. The ABTS radical cation (ABTS+) was produced by reacting the ABTS stock solution with 2.45 mM potassium persulfate (final concentration) and allowing the mixture to stand in the dark at room temperature for 12–16 h before use. Afterwards, the ABTS+ solution was diluted with ethanol to an absorbance of 0.7 ± 0.02 at 734 nm and equilibrated at 30°C. After adding 1.0 mL of diluted ABTS+ solution to 10 mL of each sample, the absorbance was measured at 30°C after 6 min. The results are expressed as the TEAC value (*μ*M/TE gram dw).

### 2.4. PBPK Model of the Methylxanthine Fraction in Rats

Simcyp*®* Animal software (version 18, release 1) was used to simulate the pharmacokinetic behaviour in experimental animals such as rats, mice, dogs, and monkeys. The available data in the software for the pharmacokinetic behaviour of caffeine in rats were used, and simulations were performed at the selected dose regimens using a complete PBPK distribution model.

### 2.5. Experimental Design

Rats were randomly divided into six groups of six animals each. Group 1 (control group) received 1 mL of physiological saline orally by gavage for 17 consecutive days. Rats in groups 2 and 3 were administered 1 mL of the methylxanthine fractions at two different doses (5 mg/kg and 1 mg/kg, respectively) orally for 17 days. Groups 4 and 5 received 1 mL of methylxanthine fractions at two different doses (5 mg/kg and 1 mg/kg, respectively) orally for 17 days and doxorubicin intraperitoneally (10 mg/kg, two doses) on the 15^th^ and 17^th^ days (cumulative dose: 20 mg/kg) 47 min after the MXB dose. Rats in group 6 (DOX group) received 1 mL of saline orally for 17 days and doxorubicin intraperitoneally (10 mg/kg body weight, two doses) on days 15 and 17 (cumulative dose: 20 mg/kg). The experimental protocol is shown in Figure 1.

During the treatment period, one rat in the DOX group died after the first intraperitoneal injection of *doxorubicin*. No deaths were observed in the other groups.

Twenty-four hours after the last DOX injection, the animals were weighed and anaesthetized with diethyl ether, and blood samples were collected from rats in all groups. Plasma was separated by centrifugation at 6000 r/min for 5 min and frozen at -20°C for estimation of the biochemical parameters. After that, the rats were sacrificed, and the hearts and kidneys were harvested and washed with ice-cold saline. Then, the organs were fixed in 10% neutral buffered formalin for histological analysis.

### 2.6. Assessment of Serum Markers for Cardio- and Nephrotoxicities

Serum creatinine, uric acid, and urea concentrations as well as serum enzyme levels (creatinine kinase (CK), creatinine kinase MB fraction (CK-MB), aspartate aminotransferase (AST), and lactate dehydrogenase (LDH)) and electrolytes (Na^+^, K^+^, and Cl^−^) were analysed using assay kits. The analyses was performed according to the instructions provided with the corresponding enzyme kit with commercially available biochemical reagents on a Cobas® 6000 analyser (F. Hoffmann-La Roche Ltd.) in a licensed laboratory in Varna. Information on the methods of analysis used is available on the site (https://usdiagnostics.roche.com/en/core_laboratory/instrument/cobas-6000-analyser-series.html # menu).

### 2.7. Histological Assessment of Cardiac and Renal Damage

The left and right ventricles of the hearts, as well as the kidneys, were fixed in 10% neutral formalin, embedded in paraffin, separated into 4-6 *μ*m thick slices using a rotary microtome, and stained with haematoxylin and eosin (H&E). A minimum of six fields from each renal section were examined, and an observer blinded to the animal treatment determined the severity of the changes. All sections were evaluated for structural changes under a Leica DM1000 LED light microscope and a Leica MC120 HD camera (Leica Microsystems AG, Wetzlar, Germany) and were captured at 200x or 400x magnification using software.

### 2.8. Statistical Analysis

All results are expressed as the arithmetic mean ± standard deviation (SD). GraphPad Prism 8.01 software (GraphPad Software, USA) was used to plot the graphs and for statistical analyses. Differences between groups were analysed using one-way ANOVA followed by Tukey's post hoc test. Six replicates were used for each different dose, and a *p* value < 0.05 was considered a statistically significant difference.

## 3. Results

### 3.1. Antioxidant Activity of the Methylxanthine Fraction Isolated from Bancha Tea Leaves

The antioxidant activity results are presented in Table 1.

As seen in the table, the methylxanthine fraction exhibited significant antioxidant activity, which could be utilized for further research.

### 3.2. Simulation of the Pharmacokinetic Behaviour of the Methylxanthine Fraction in Rats

It was hypothesized that the pharmacokinetic behaviour of methylxanthines would be similar to that of caffeine. Based on this and the available physicochemical and pharmacokinetic data on caffeine in rats from the software Simcyp*®* Animal (version 18, release 1), an experimental design was simulated using the higher dose of 5 mg/kg methylxanthine fraction to determine the plasma and tissue peaks (heart and kidney) and to test for the expected protective effects. A full PBPK distribution model was used for this purpose, and the simulation results are shown in Table 2 and Figure 2.

As seen from the graph and the table, the two richly supplied blood organs—the heart and kidneys—receive a significant amount of the administered methylxanthine fraction. Peaks in tissue concentrations are reached after nearly 47 min.

### 3.3. Changes in Biochemical Markers of Cardiac and Renal Damage

Cardio- and nephrotoxicity models induced by the cumulative dose of doxorubicin (20 mg/kg) show significant differences in the biochemical parameters (that are not shown in the figures) compared to the control group (*p* < 0.001, receiving physiological solution only), indicating cardiac and renal tissue damage. *Bancha* methylxanthine administration alone did not lead to significant changes compared to the control group (*p* = 0.573). However, the simultaneous treatment of *doxorubicin* and methylxanthines demonstrated a dose-dependent reduction in the serum levels of the biochemical parameters tested, which indicates a decrease in cardiac (*p* < 0.05 for CK, CK-MB, and AST; *p* < 0.01 for LDH) and renal (*p* < 0.01 for uric acid; *p* < 0.05 for creatinine and BUN) tissue damage compared to rats treated with doxorubicin alone. Statistically significant changes in the cardiac marker troponin I (cTnI) were not detected, and its levels were not elevated in the control, treatment, or model groups. Serum levels of electrolytes (Na^+^, K^+^, and Cl^−^) were also not significantly altered. Tables 3 and 4 and Figures 3 and 4 show the influence of methylxanthines isolated from *Bancha* tea leaves on the biochemical parameter serum levels for cardio- and nephrotoxicities.

### 3.4. Effects on the Histological Parameters of Cardio- and Nephrotoxicities

Examination of haematoxylin-eosin-stained longitudinal sections of the control group (group 1) revealed a normal histological structure of the ventricular myocardium (Figure 5(a)) with branched and transverse striated muscular fibres with central oval nuclei. In contrast, rats treated with doxorubicin alone (group 6) showed significant histological changes (Figure 5(b)) including disrupted myofibril architecture, myocyte disorganization, cytoplasmic fading, and pyknotic nucleus formation. On the other hand, pretreatment with methylxanthines at the dose of 5 mg/kg (Figure 5(c)) led to an almost normal myocardial structure with very limited mononuclear infiltration of the interstitium and a marked reduction in collagen fibres between cardiac myocytes compared to the *doxorubicin* group.

Histological examination of the renal tissue in the control group rats showed normal architectures of the renal glomeruli and tubules (Figure 6(a)). The *doxorubicin* group (Figure 6(b)) showed significant glomerular and tubular disorders. Total collapse of the glomeruli with necrotic changes in the epithelial tubular cells was observed. Both groups, after pretreatment with *Bancha* methylxanthines (5 mg/kg and 1 mg/kg) (Figures 6(c) and 6(d), respectively) demonstrated significant resistance to the deleterious effects of *doxorubicin*. The lesions were mainly in the cortical area. At the higher dose of methylxanthines, there was a significant decrease in the morphological changes caused by doxorubicin exposure.

## 4. Discussion

In the first part of our study, we assessed the antioxidant potential of the isolated methylxanthine fraction from *Bancha* using DPPH and ABTS assays. Both methods are widely used for determining the antioxidant activity of natural compounds [15, 16]. The *in vitro* observed significant antioxidant activity of methylxanthines (Table 1) has also been confirmed by other authors *in vitro* and *in vivo* [17, 18]. The most studied methylxanthine is caffeine, which suppresses major reactive oxygen radicals (e.g., hydroxyl radicals, peroxyl radicals, and singlet oxygen). As noted above, in our previous study, HPLC analysis of the methylxanthine fraction showed 88.11% caffeine, 0.42% theobromine, and no theophylline content [13], whereby our assumptions were made that the properties of this fraction would be similar to that of caffeine, and this could be used for amelioration of doxorubicin-induced oxidative stress. In order to verify this hypothesis, we conducted *in vivo* experiments with *doxorubicin*-induced cardio- and nephrotoxicities in rats. In our previous study, methylxanthines isolated from *Bancha* showed synergistic effects with doxorubicin against the triple-negative breast cancer cell line MDA-MB-231 [19], which suggests that this combination may simultaneously increase therapeutic effects and reduce adverse effects.

Before conducting animal experiments, based on the abovementioned assumptions, simulations using Simcyp® Animal software to examine the pharmacokinetic behaviour of the methylxanthine fraction in rats was performed. The caffeine content in one cup of Bancha tea, as in most caffeinated beverages, is not constant and varies; therefore, based on our previous research [20], doses approaching the lower 1 mg/kg level and upper 5 mg/kg level were selected. The simulation results with the higher concentration presented in Table 2 and Figure 2 indicate peak plasma concentrations at the 38^th^ minute and peak concentration in the tissues of interest (heart and kidney) at the 47^th^ min. Therefore, administration of doxorubicin in groups pretreated with methylxanthine was 47 min after the last treatment, suggesting maximum tissue concentration of the protective agent.

In our study, lower administered doses (1 mg/kg) of the *Bancha*-isolated methylxanthine fraction led to a decrease in the biochemical markers of toxicity in the heart and kidney, but without a statistically significant difference compared to the doxorubicin group (*p* > 0.05), except for lactate dehydrogenase (LDH) and uric acid (*p* < 0.05). In contrast, the higher dose used (5 mg/kg) led to a statistically significant (*p* < 0.05) reduction of all the abovementioned biochemical markers, which was supported by the histological studies. We assumed that the possible mechanism of action of Bancha methylxanthines is due to their significant antioxidant properties, supporting the hypothesis that oxidative stress caused by ROS is the major reason for doxorubicin cardiac and renal toxicities [21].

We found no statistically significant (*p* > 0.05) changes in the studied electrolytes (Na^+^, K^+^, and Cl^−^), which was also previously reported by other authors in other animal models [22], although others have reported significant changes [23]. At this stage, we have no explanation for why cardiac troponin I (cTnI) levels were not elevated, as its values were <0.20 ng/mL in the control and MXB pretreatment groups as well as in the doxorubicin group.

No data were found regarding the cardioprotective activity of the selected methylxanthine fractions or their components in the literature. In contrast, an increase in cardiotoxicity was reported when the major component in the methylxanthine fraction (caffeine) was used [24, 25]. This is probably due to the mechanism of action of methylxanthines associated with the blockade of adenosine receptors. Adenosine is released during ischaemia and has a protective effect on the heart by acting on two subtypes of adenosine receptors—A_1_ and A_3_ [26]. In addition, *caffeine* stimulates ryanodine receptors (RyRs) and leads to an increase in intracellular calcium, which contributes to the depolarization and contractility of cardiomyocytes [27]. In the cited sources, Dunnick et al. (2007) and Howden et al (2005), *caffeine* was administered concomitantly with *ephedrine* to induce cardiotoxicity in rodents. In addition, the doses used in these studies were 15-30 mg/kg and 30 mg/kg, respectively. In our studies, the doses were significantly lower, and if we recalculate the *caffeine* content at the highest dose used in the current study based on HPLC fraction analysis, then the caffeine dose would be approximately 4.4 mg/kg. It should be noted that this fraction contains other substances that have not been analysed at this stage, but it is assumed that they also participate in the biological activity. A literature review showed that cardioprotective activity has been identified for extracts of coffee or green tea, but the authors mainly attributed this activity to the catechin and polyphenol components [28, 29].

Information in the scientific literature mainly supports the nephroprotective effects of methylxanthines [30, 31]. For example, Potier et al. (1997) reported that methylxanthine derivatives (caffeine, theophylline, and pentoxifylline) showed protective effects on cyclosporine A-induced glomerular contraction in isolated glomeruli and cultured rat mesangial cells. Benoehr et al. (2005) used theophylline in a randomized, single-blinded, placebo-controlled human trial for nephroprotection with cisplatin-based chemotherapy. The authors concluded that prophylactic theophylline administration may prevent renal function impairment in cisplatin-based chemotherapy with respect to the glomerular filtration rate (GFR). However, other clinical studies have shown that theophylline has no such nephroprotective effect [32].

We acknowledge that this study has some limitations. After identifying certain substances, we did not find a proper match for a positive control. Moreover, recently published studies did not include positive controls [33, 34]. Toxicity studies were not performed since methylxanthines have been well studied, and the doses used in the present study are significantly lower than the lethal doses of caffeine, theobromine, and theophylline in rats. The objective of our future studies is to clarify the heart and kidney tissue oxidative stress reduction inflicted by methylxanthines and to precisely explain the mechanisms involved in the observed organ-protective effects.

## 5. Conclusion

The methylxanthine fraction isolated from *Bancha* has shown encouraging results in terms of its combined potential with conventional chemotherapeutic agents such as *doxorubicin*. On the one hand, *in vitro* synergistic effects with *doxorubicin* have been demonstrated with respect to methylxanthine fraction coadministration to breast cancer cells, and on the other hand, the methylxanthine fraction has shown the potential to reduce the major limiting factors from the usage of *doxorubicin*, namely, cardio- and nephrotoxicities, in *in vivo* rat models.

## Figures and Tables

**Figure 1:** Experimental protocol.

**Figure 2:** Generation of full PBPK model after simulation of per oral administration of 5 mg/kg MXB using Simcyp Animal software.

**Figure 3:** Changes in the biochemical markers for cardiotoxicity on pretreatment with *Bancha* methylxanthines at doses of 5 mg/kg (group 4) and 1 mg/kg (group 5) compared to the doxorubicin model (group 6). The values are presented as mean ± SD. One-way ANOVA test was performed for comparison between the groups. ^∗^*p* < 0.5 and ^∗∗^*p* < 0.01 compared to the model.

**Figure 4:** Changes in the biochemical markers for nephrotoxicity on pretreatment with *Bancha* methylxanthines at doses of 5 mg/kg (group 4) and 1 mg/kg (group 5) compared to the *doxorubicin* model (group 6). The values are presented as mean ± SD. One-way ANOVA test was performed for comparison between the groups. ^∗^*p* < 0.5 and ^∗∗^*p* < 0.01 compared to the model.

**Figure 5:** Photomicrographs of muscle sections of left ventricular chambers stained with H&E ×400. (a) Control; normal myofibrilar architecture. (b) *Doxorubicin*-treated group (cumulative dose: 20 mg/kg); disorganization of cardiac muscle fibres (arrow left), cytoplasmic fading, and pyknotic nucleus formation (arrow above) and myofibril ruptures (arrow right). (c) A group pretreated with MXB (5 mg/kg); ameliorated myofibrilar disorganization.

**Figure 6:** Photomicrographs of renal cortex stained with H&E ×400. (a) Control; normal structure of nephrons. (b) *Doxorubicin*-treated group (cumulative dose: 20 mg/kg); damaged tubular cells (arrow left) and total collapse of glomeruli (arrow right). (c, d) Groups pretreated with MXB 5 mg/kg and 1 mg/kg; the both groups show less damage of kidney tissue. The lesions are mainly in the cortical area.

**Table 1:** Antioxidant activity of methylxanthine fraction isolated from *Bancha* (MXB) determined by two methods—DPPH and ABTS and expressed as millimole trolox equivalents (mM TE) on gram dry extract (DE).

	DPPH mM TE/g *DE* ± *SD*	ABTS mM TE/g *DE* ± *SD*
Methylxanthine fraction isolated from *Bancha* (MXB)	592.71 ± 1.67	3326.2 ± 1.03

**Table 2:** *C*_max_, *t*_max_, and AUC values in rat plasma, heart, and kidney after simulation of per oral administration of 5 mg/kg MXB using Simcyp Animal software.

	*C*_max_ (mg/L)	*t*_max_ (h)	AUC (mg·h/L)
Plasma concentrations	4.94	0.64	13.76
Heart concentrations	3.04	0.79	8.62
Kidney concentrations	2.98	0.79	8.46

**Table 3:** Effects of *Bancha* methylxanthine administration at doses of 5 mg/kg and 1 mg/kg on CK, CK-MB, LDH, and AST enzyme activities in *doxorubicin*-induced cardiotoxicity (cumulative dose: 20 mg/kg).

Groups	Creatinine kinase (CK) (U/L)	Creatinine kinase MB fraction (CK-MB) (U/L)	Lactate dehydrogenase (LDH) (U/L)	Aspartate aminotransferase (AST) (U/L)
Group 1: control	324 ± 14	22.3 ± 1.6	209.63 ± 19.6	89.87 ± 9.87
Group 2: 5 mg/kg (p.o.) MXB	304 ± 9.7	24.7 ± 3.6	155.63 ± 7.6	78 ± 5.7
Group 3: 1 mg/kg (p.o.) MXB	311 ± 9.6	23.7 ± 3.6	164.7 ± 5.8	69.7 ± 6.7
Group 4: 5 mg/kg (p.o.) MXB+doxo 20 mg/kg (i.p.)	856.8 ± 69.4	34 ± 5.7	325 ± 32.6	254.8 ± 46.9
Group 5: 1 mg/kg (p.o.) MXB+doxo 20 mg/kg (i.p.)	987.65 ± 121.4	37 ± 4.6	444 ± 43.7	584 ± 32.8
Group 6: doxo 20 mg/kg (i.p.)	1260 ± 80.1	47.8 ± 7.8	633.11 ± 32.4	687.23 ± 22.35

**Table 4:** Effects of *Bancha* methylxanthine administration at doses of 5 mg/kg and 1 mg/kg on serum levels of urea, creatinine, and uric acid in doxorubicin-induced nephrotoxicity (cumulative dose: 20 mg/kg).

Groups	Urea (BUN) (mmol/L)	Creatinine (*μ*mol/L)	Uric acid (*μ*mol/L)
Group 1: control	6.3 ± 0.8	37.71 ± 3.6	32.7 ± 2.6
Group 2: 5 mg/kg (p.o.) MXB	7.4 ± 0.54	38.64 ± 2.7	36.6 ± 3.43
Group 3: 1 mg/kg (p.o.) MXB	7.7 ± 0.96	35.75 ± 2.8	34.6 ± 1.7
Group 4: 5 mg/kg (p.o.) MXB+doxo 20 mg/kg (i.p.)	7.88 ± 1.1	42.54 ± 5.98	55.2 ± 4.32
Group 5: 1 mg/kg (p.o.) MXB+doxo 20 mg/kg (i.p.)	9.87 ± 1.6	59.3 ± 2.8	98.8 ± 6.5
Group 6: doxo 20 mg/kg (i.p.)	11.11 ± 0.8	62.45 ± 5.6	247.41 ± 25.4

## Data Availability

The data used to support the findings of this study are available from the corresponding author upon request.
